# Factors Affecting Adenoma Risk Level in Patients with Intestinal Polyp and Association Analysis

**DOI:** 10.1155/2022/9479563

**Published:** 2022-01-15

**Authors:** Ying Dai, Weimin Chen, Xuanfu Xu, Jianqing Chen, Wenhui Mo, Yiming Chen, Shuqi Xu

**Affiliations:** Department of Gastroenterology, Shidong Hospital of Yangpu District, Shanghai 200438, China

## Abstract

**Objective:**

To explore the factors affecting the adenoma risk level in patients with intestinal polyp and association.

**Methods:**

The clinical data of 3,911 patients with intestinal polyp treated in our hospital from January 2018 to January 2021 were retrospectively analyzed, all patients accepted the histopathological examination, their risk of suffering from adenoma was evaluated according to the results of pathological diagnosis, and relevant hazard factors affecting adenoma risk level in them were analyzed by multifactor logistic regression analysis.

**Results:**

The results of multifactor logistic analysis showed that male gender, age ≥60 years, number of polyps >3, diameter ≥2 cm, onset at colon, and physiologically tubulovillous adenoma were the hazard factors causing high-grade adenoma risk in patients with intestinal polyp.

**Conclusion:**

There are many risk factors causing high-grade adenoma in patients with intestinal polyp, and therefore, the screening for high-risk population shall be enhanced to reduce the potential of carcinomatous change in such patients.

## 1. Introduction

Intestinal polyps refer to protrusion lesions on the surface of the intestinal mucosa that protrude into the lumen and belong to an abnormally growing tissue that can occur anywhere in the intestine, with colonic polyps, rectal polyps, and colorectal polyps being the common types [1]. Adenomatous and nonadenomatous polyps are classified on the basis of pathologic biopsies, and the former is more prone to atypical hyperplasia and malignant change and, when underappreciated, may progress to colorectal cancer [2, 3]. Colorectal cancer refers to cancers of epithelial origin in the large intestine, which often presents clinically with abdominal pain, bloating, and reduced intestinal function, and with the progression of the disease, can also invade surrounding tissues or organs, causing urinary urgency and hematuria. Foreign studies have shown that [4] 25%–45% of patients with intestinal polyps will relapse at 3–5 years, with a cumulative recurrence rate of 52.3% at 1 year and 70.8% at 2 years. Intestinal polyps mainly grow in the rectum and sigmoid colons, which present clinical symptoms such as intestinal bleeding, abdominal pain, and abdominal distension, seriously affecting the quality of life of patients. Investigations have revealed [5, 6] that intestinal polyps are the most predominant precancerous lesions of colorectal cancer; thus, it is particularly important for early detection, treatment, and follow-up of intestinal polyps. According to research findings, intestinal carcinomatous change is related to the size, pathology, age, and other factors of adenomas, and its carcinogenesis time is about 10–15 years, which provides the temporal feasibility for early intervention in the malignant transformation of adenomatous polyps, and therefore, it is important to summarize the risk factors for the development of a high-grade risk of adenoma in patients with various types of intestinal polyps [7–9]. The current rule of colon polyp—adenoma—carcinomatous change has been generally accepted, so attention shall be paid to patients who have adenomatous polyps, and early detection and resection can reduce the risk of colorectal cancer to some extent. So far, there are many factors associated with the carcinogenesis of polyps, including drinking, smoking, dietary habits, and family heredity, but the specific mechanism is still not clear with diversed conclusions [10]. Hence, the risk factors causing high-grade adenomas in patients with polyps were explored herein, with the results reported as follows.

## 2. Data and Methods

### 2.1. General Information

The clinical data of 3,911 patients pathologically diagnosed with intestinal polyps and treated in our hospital from January 2018 to January 2021 were retrospectively analyzed, and the study met the World Medical Association Declaration of Helsinki [11]. Exclusion criteria for the patients: (1) familial intestinal polyposis, (2) history of colon surgery, (3) failure to complete polyp treatment, (4) ulcerative colitis, and (5) malignancy. The research technical route is shown in Figure 1.

### 2.2. Methods

#### 2.2.1. Obtaining Clinical Data

It was a retrospective observational study. Through reviewing and screening the electronic medical record system of our hospital, the clinical data of patients diagnosed with intestinal polyp, colonic polyp, multiple colonic polyp, rectal polyp, multiple rectal polyp, colorectal polyp, and multiple colorectal polyp and discharged from our department of digestive medicine were collected. By tracking their medical records, whether there was medical advice on return visit in the discharge abstract, the return visit records in the electronic out-patient medical records after discharge, and the colonoscopy results during return visit in the colonoscopy examination database were checked. The patients who did not return for subsequent examination were contacted via telephone and asked whether they had went to other hospitals as schedule for colonoscopy.

#### 2.2.2. Collected Information

The collected information includes patients' name, age, gender, BMI value, medical history, and number, size, position, shape, and pathological type of polyp.

#### 2.2.3. Histopathological Evaluation

After excision of colonic adenoma under the endoscope, the specimens were processed with routine method and stained with hematoxylin and eosin. The pathologic structure and other conditions of the specimens were evaluated according to the criteria of the World Health Organization [12].

### 2.3. Statistical Methods

In this study, the data processing was conducted with the professional statistic software SPSS 24.0, the picture drawing software was GraphPad Prism 7 (GraphPad Software, San Diego, USA), the relevant risk factors causing high-grade adenoma in patients with intestinal polyp were analyzed by multifactor logistic analysis, and differences were considered statistically significant at *P* < 0.05.

## 3. Results

### 3.1. Basic Condition of Patients

Analysis of the clinical data of the study subjects revealed that most patients were male, elderly, and complicated with hypertension, and the pathology was dominated by villous tubulation (Table 1).

### 3.2. Multifactor Retrospective Analysis on Occurrence of High-Grade Adenoma

Age ≥60 years, male gander, number of polyps >3, diameter ≥2 cm, onset at the colon, and pathologically tubulovillous adenoma were the independent risk factors causing high-grade adenoma in patients with intestinal polyp (Table 2).

### 3.3. Correlation Analysis on Occurrence of High-Grade Adenoma in Patients

Figure 2 shows the correlation analysis on occurrence of high-grade adenoma in patients.

### 3.4. Comparison of Areas under Curve among Various Indicators

The area under curve of pathologically tubulovillous adenoma was higher than that of other single indicators (Table 3).

### 3.5. Comparison of Sensitivity and Specificity among Various Indicators

Pathologically tubulovillous adenoma had the highest sensitivity, and onset at colon had the highest specificity (Table 4).

## 4. Discussion

Clinically, polyp lesions that protrude on the surface of the colorectal mucosa and of undetermined pathological type are collectively referred to as intestinal polyps [13, 14], which can be specifically classified as adenomatous polyps versus nonadenomatous polyps, and based on the pathological diagnostic findings, adenomatous polyps can be further classified as colonic inflammatory polyps and tubular adenomas of the colon [15]. Adenomatous polyps are currently recognized as the most important precancerous lesions of colorectal tumors, with a carcinogenesis rate of up to 9.7% and the incidence gradually increasing with age [16–18]. High-grade adenoma generally grows in the colonic or rectal mucosa, individually in the small intestine; as the tumor increases in size and becomes solid in texture, it severely affects defecation and causes inconvenience to the patients' life. Therefore, it is important for early prevention of colorectal cancer by investigating the risk factors for the development of high-grade adenomas from intestinal polyps.

This study has a significant guiding value for primary prevention and early diagnosis of colorectal cancer by carrying out retrospective analysis and adopting multivariate logistic analysis on risk factors affecting the adenoma risk grade in patients with intestinal polyps, aiming to fully understand the rules of occurrence and development of intestinal polyps and to implement early intervention [19, 20]. In this study, gender was found to be an independent risk factor for high-grade adenoma in patients with intestinal polyps, but this indicator is somewhat controversial among studies; some reported [21] that the incidence of high-grade adenoma in male patients with intestinal polyps was significantly higher than that in female patients, which might be due to their bad living habits such as drinking and smoking [22]. This study found a link between the occurrence of high-grade adenomas and gender, but such viewpoint remains to be proved by epidemiological studies with larger samples. In addition, this study confirmed that pathological villous tubulation was also an independent risk factor for inducing high-grade adenomas in patients with intestinal polyps. Gupta et al. [23] found that the more villous component in intestinal polyps, the higher the likelihood of carcinogenesis, so it was speculated that the mechanism might be that villous tubular structure increased the surface area of adenoma to some extent, which, combined with the faster growth rate of villous tubular adenoma, resulted in its lower apoptosis rate than other pathological types. In addition, it has been found that the risk of developing high-grade adenoma rises with age, so annual colonoscopy in patients older than 50 years is recommended to increase the clinical detection rate of colonic neoplasia, and the higher the number and diameter of polyps, the higher the risk of developing carcinoma. Also, some scholars [24] concluded that polyps with larger diameter are more prone to progressive histopathological changes and therefore cannot be ignored. This study found that polyps ≥2 cm in diameter are a risk factor for the development of high-grade adenomas, so when undergoing electronic colonoscopy, every polyp should be biopsied whenever possible to avoid omission [25]. By plotting the ROC curve in this study, the correlation between each risk factor and high-grade adenoma was analyzed, and it was found that the area under the curves for factors such as pathological tubulovillous adenoma and onset at colon was larger, and therefore, these factors could provide a theoretical basis for clinical diagnosis and prevention of high-grade adenoma. Due to the limitations of this study, the study subjects were only the patients of our region and did not include those from other provinces and ethnic minorities, so it may cause the results to be influenced by small sample size, geographical culture, and ethnic differences. Therefore, further improvement is required.

## Figures and Tables

**Figure 1:** Research technical route.

**Figure 2:** Correlation analysis on occurrence of high-grade adenoma in patients.

**Table 1:** General condition of patients with intestinal polyp.

Item	Number of cases	Proportion (%)
Male	2,245	57.40

BMI grade		
Normal	2,565	65.58
Underweight	134	3.43
Overweight	1,212	30.99
Mean height (cm)	169.23 ± 6.17	—
Mean weight (kg)	64.51 ± 12.21	—

Age cohort		
18–26 years	5	0.13
27–48 years	211	5.40
49–60 years	778	19.89
≥60 years	2,917	74.58

Underlying disease		
Hypertension	2,069	52.90
Diabetes	697	17.82
Coronary heart disease	309	7.90
Cerebral infarction	270	6.90
History of tumor	566	14.47
Smoking	1,251	31.99
Drinking	464	11.86

Number of polyps		
≤2	1,527	39.04
>3	2,384	60.96

Diameter		
≤0.5 cm	1,176	30.07
0.6–1.2 cm	2,217	56.69
1.3–1.9 cm	165	4.22
≥2.0 cm	353	9.03

Pathogenic site		
Cecum	76	1.94
Transverse colon	687	17.57
Descending colon	842	21.53
Sigmoid colon	708	18.10
Rectum	413	10.56
Polyp	240	6.14
Ascending colon	945	24.16

Pathology		
Hyperplasia	463	11.84
Tubular	425	10.87
Villus	373	9.54
Tubulovillous	1,026	26.23
Serrated	469	11.99
High-grade tubular adenoma	381	9.74
High-grade tubulovillous adenoma	774	19.79

**Table 2:** Multifactor logistic analysis on occurrence of high-grade adenoma in patients with intestinal polyp.

Item	HR	95% CI	*P* value
Age (≥60 years)	1.014	0.725–1.352	0.035
Gender (male)	0.826	0.426–1.124	0.042
Smoking	1.237	0.936–1.426	0.526
Drinking	0.936	0.735–1.351	0.263
Combined underlying diseases	1.127	0.936–1.327	0.152
Number of polyps >3	0.835	0.726–1.125	0.016
Diameter ≥2 cm	1.217	0.826–1.526	0.025
Onset at the colon	1.035	0.721–1.361	0.009
Pathologically tubulovillous adenoma	1.236	0.923–1.473	<0.001

**Table 3:** Comparison of areas under curve of various indicators.

Test result variable	Area	S.E.^a^	Asymptotic sig.^b^	Asymptotic 95% CI	
				Lower limit	Upper limit
Male gender	0.830	0.044	0.000	0.745	0.915
Age ≥60 years	0.810	0.046	0.000	0.721	0.899
Number of polyps >3	0.860	0.040	0.000	0.781	0.939
Onset at colon	0.900	0.035	0.000	0.832	0.968
Pathological tubulovillous adenoma	0.910	0.033	0.000	0.845	0.975
Diameter ≥2 cm	0.810	0.046	0.000	0.721	0.899

**Table 4:** Diagnostic results of various indicators.

Indicator	Male gender	Age ≥60 years	Number of polys >3	Onset at colon	Pathologically tubulovillous adenoma	Diameter ≥2 cm
Sensitivity (%)	89.29	83.33	86.21	89.29	92.59	87.72
Specificity (%)	83.33	86.21	89.29	92.59	90.91	80.65

## Data Availability

The data used to support the findings of this study are available from the corresponding author upon request.
